The article "Progress of genome wide association study in domestic animals" was retracted in 2013. Reason: plagiarism.

# Progress of genome wide association study in domestic animals

**DOI:** 10.1186/2049-1891-3-26

**Published:** 2012-08-22

**Authors:** Hui Zhang, Zhipeng Wang, Shouzhi Wang, Hui Li

**Affiliations:** 1 Key Laboratory of Chicken Genetics and Breeding, Ministry of Agriculture, Harbin, 150030, People's Republic of China; 2 College of Animal Science and Technology, Northeast Agricultural University, Harbin, 150030, People's Republic of China

**Keywords:** Domestic animals, Genome wide association study (GWAS), Quantitative trait loci (QTL), Single-nucleotide polymorphism (SNP)

## Abstract

Domestic animals are invaluable resources for study of the molecular architecture of complex traits. Although the mapping of quantitative trait loci (QTL) responsible for economically important traits in domestic animals has achieved remarkable results in recent decades, not all of the genetic variation in the complex traits has been captured because of the low density of markers used in QTL mapping studies. The genome wide association study (GWAS), which utilizes high-density single-nucleotide polymorphism (SNP), provides a new way to tackle this issue. Encouraging achievements in dissection of the genetic mechanisms of complex diseases in humans have resulted from the use of GWAS. At present, GWAS has been applied to the field of domestic animal breeding and genetics, and some advances have been made. Many genes or markers that affect economic traits of interest in domestic animals have been identified. In this review, advances in the use of GWAS in domestic animals are described.

## Introduction

The concept and means to identify genes related to complex traits at the genome-wide level can be traced back to the 1990s. Mapping of quantitative trait loci (QTL) was the preferred approach to detect genetic variation for economically important traits at the genome-wide level. To date, thousands of QTLs for numerous traits have been reported (http://www.animalgenome.org/QTLdb/). However, most of these reported QTLs were detected using microsatellite markers with low map resolution and the confidence interval (CI) covers more than 20 cM [1], even a whole chromosome [2]. Therefore, it is difficult to detect the important genes for traits of interest based on the information. The identification of causal mutations that underlying QTLs has been challenging in domestic animals. The genome wide association study (GWAS) is a new technique for the identification of causal genes for important traits in livestock. The GWAS uses sequence variations (mainly single nucleotide polymorphisms, SNPs) in the whole genome, together with the phenotype and pedigree information, to perform association analysis and to identify genes or regulatory elements that are important for the traits of interest. GWAS has become feasible in humans as well as in domestic animals as a result of the development of large collections of SNPs and the development of cost-effective methods for large-scale SNP analysis. Compared with traditional QTL mapping strategies, GWAS confers major advantages both in the power to detect causal variants with modest effects and in defining narrower genomic regions that harbor causal variants [3]. GWAS is an ideal technique to discover the major genes for complex traits and is a novel way to study the genetic mechanism of complex traits. In this paper, we reviewed the progress of GWAS in domestic animals.

## Progress of GWAS in domestic animals

GWAS was first used in the analysis of human disease and great progress was made. GWAS was extended to the field of domestic animal genetics and breeding when genomic sequences were available for several domestic species and large numbers of SNPs were discovered as a by-product of sequencing or in subsequent re-sequencing. There are many kinds of commercial SNP chip available for cattle (50,000 SNPs; Illumina BovineSNP50 BeadChip), dogs (22,362 SNPs; Illumina CanineSNP20 BeadChip), sheep (56,000 SNPs), pigs (60,000 SNPs; Illumina PorcineSNP60 BeadChip), horses (54,602 SNPs; Illimina EquineSNP50 BeadChip) and chickens (60,000 SNPs; Illumina ChickenSNP60 BeadChip). Although the application of GWAS to domestic animals has only occurred relatively recently, there have been a series of results reported, especially from the analysis of the genetic mechanisms of quantitative traits.

An assumption made in the analysis of GWAS is that significant associations can be detected because the SNPs are in linkage disequilibrium (LD) with the causative mutations for the traits of interest. The high density of SNP markers in the chip used in GWAS was sufficient to identify the LD between SNP markers and causative mutations. During the past few years, several examples of successful GWAS in domestic animals, including cattle, pigs, horses, dogs, sheep and chickens, have been reported (Table 1).

**Table 1:** Summary of reported GWAS on domestic animals

**No.**	**Trait**	**Chip**	**Animal**	**Method**	**Significant level**	**Result**	**Ref**
1	Milk yield	50K	62,343 Holstein Friesian cows sired by 798 sires	Mixed linear models	*P <* 0.001	Identified 362 significant SNPs	[4]
2	Milk yield	50K	767 Holstein bulls	Single and Multiple trait regression analysis	*P <* 0.001	Identified 169 significant SNPs	[5]
3	Milk yield	50K	2,093 Chinese Holstein from the Holstein cattle farms in Beijing, China	Single locus regression analysis	Bonferroni *P <* 0.05 level	Identified 105 significant SNPs including two SNPs located close to the *DGAT1* gene (160bp apart) and within the *GHR* gene, respectively	[6]
4	Milk yield	50K	1,039 bulls with pedigree information from Danish Jersey cattle	Regression analysis	Bonferroni correction *P <* 1.5e^−6^	Identified 98 significant SNPs	[7]
5	Milk quality traits	50K	780 Holstein sons of 142 sires	Bayesian analysis (BayesA)	*P ≤* 0.001	Identified 73-461 significant SNPs (depending on trait)	[8]
6	Milk quality traits	50K	3,356 Japanese Black cattle from Yamagata Prefecture	GRAMMAR-CG method	Bonferroni correction *P <* 1.28e^-6^ (5%); *P <* 2.57e^-7^ (1%)	Identified 32 significant SNPs mainly in region of 49-55 Mb on BTA19 containing *FASN* gene	[9]
7	Milk quality traits	50K	1,905 Dutch Holstein Friesian cows from 398 commercial farms throughout the Netherlands	Two step single SNP association analysis using general linear model and animal model	FDR < 0.05	Identified 54 significant regions mainly on BTA14, 19, and 26 containing *ABCG2*, *PPARGC1A*, *ACSS2*, *DGAT1*, *ACLY*, *SREBF1*, *STAT5A*, *GH*, *FASN*, *SCD1*and *AGPAT6*	[10]
8	Milk quality traits	50K	1,912 Holstein-Friesian cows from 398 commercial herds throughout the Netherlands	General linear model	FDR <0.01	Identified several important regions mainly on BTA5, 6, 11 and 14	[11]
9	Fertility trait	10K	10 low-fertility and 10 high-fertility bulls of Pure Holstein	Regression analysis	*P <* 0.01	Identified 97 significant SNPs including one SNP in Integrin beta 5 gene	[12]
10	Fertility trait	50K	267 Holstein cows	Generalized linear mixed model	*P <* 0.05	Identified 27 significant SNPs	[13]
11	Fertility trait	50K	2,531 Danish and Swedish Holstein bulls	Mixed model analysis	Bonferroni correction *P <* 2.16e^-5^ (BTA1); *P <* 7.41e^-5^ (BTA28)	Identified 74 significant SNPs mainly on BTA 3, 5, 10, 13, 19, 20, and 24	[14]
12	Fertility trait	50K	2,062 Danish and Swedish Holstein bulls	Mixed model analysis	Bonferroni correction *P <* 2.16e^-5^ (BTA1); *P <* 7.41e^-5^ (BTA28)	Identified several important regions on BTA4, 6, 12, 18, 20, and 25	[15]
13	Growth trait	50K	150 sires representing 7 breeds including Angus, Charolais, Gelbvieh, Hereford, Limousin, Red Angus and Simmental	ANOVA test	FDR < 0.01	Identified 231 significant SNPs	[16]
14	Growth trait	10K; 50K	852 steers from 7 different pure breeds including Angus, Murray Grey, Shorthorn, Hereford, Brahman, Santa Gertrudis and Belmont Red	Regression analysis	*P* <0.001	Identified 75 significant SNPs mainly on BTA3, 5, 7, and 8	[17]
15	Meat quality and carcass traits	50K	940 Beef cattle	Regression analysis	*P* <0.001	Identified 87 significant SNPs for meat quality traits and 127 significant SNPs for carcass traits	[18]
16	Classical bovine spongiform encephalopathy (BSE)	50K	Holstein cows including 143 BSE affected (case) and 173 unaffected (control) collected in Southern England	Chi-square test	*P <* 5e^-5^	Identified one SNP on chromosome 1 at 29.15 Mb and another locus on chromosome 14	[19]
17	Bovine Tuberculosis (TB)	50K	14,013 Irish Holstein- Friesian cows	Regression analysis	Bonferroni correction *P <* 1.21e^-6^	Identified 3 significant SNPs in a 65kb genomic region on BTA 22 containing *SLC6A6* gene	[20]
18	Bovine Paratuberculosis	50K	Italian and American Holstein cows including Group A with 590 cases vs 600 controls and Group B with 590 cases vs 117 controls	GRAMMAR-CG method	*P <* 5e^-5^	Identified 6 significant SNPs on BTA 1, 12 and 15 and several other significant SNPs on BTA 1, 6, 7, 13, 16, 21, 23 and 25	[21]
19	Dominant White Phenotype and Bilateral Deafness	770K	Seven white and 79 spotted German Fleckvieh	General Linear Model (GLM)	-log_10_P_raw_ = 254.4; -log_10_P_Bonferroni-adjusted_ = 248.6	Identified a most significant region on BTA 22 containing *MITF* gene	[22]
20	Androstenone	60K	987 pigs divergent for androstenone concentration from a commercial Duroc- based sire line	QFAM test	FDR of q-value ≤ 0.05	Identified 37 significant SNPs mainly on SSC1 and SSC6	[23]
21	skatole levels	60K	891 pigs from a composite Duroc sire line	QFAM test	FDR of q-value ≤ 0.05	Identified 16 significant SNPs on SSC6: 0-6Mb	[24]
22	Boar taint and related sex steroids	60K	1,251 purebred Norwegian Landrace and 918 purebred Duroc male pigs	ANOVA test	*P* < 0.05	Identified g 28 regions related to boar taint	[25]
23	Boar taint and fertility traits	60K	1,533 purebred Landrace and 1,027 purebred Duroc male pigs	ANOVA test	*P* < 0.05	Identified 34 significant regions mainly on SSC1, 2, 3, 4, 7, 13, 14 and 15	[26]
24	Knobbed acrosome defect	60K	14 Finnish Yorkshire boars affected with KAD and 21 controls	Chi-square test	Permutation correction *P <* 0.0002	Identified a significant 0.7 Mb region on SSC15 containing *STK17b* and *HECW2* genes	[27]
25	Body Composition and Structural Soundness Traits	60K	412 Large White line pigs and 408 pigs from a Large White × Landrace cross	Bayes C	Bootstrap correction 0.001 < P < 0.002	Identified several important genes including *MC4R*, *IGF2*, *CHCHD3*, *BMP2* and *HOXA*	[28]
26	Fat area	60K	150 crossbred pigs [Pietrain × (German Large White × German Landrace)]	ANOVA test	*P <* 1.0e^-5^	Identified 663 important genes	[29]
27	Brown coat colour	60K	Brown pigs (n = 121) vs non-brown-coated pigs (n = 745)	Chi-square test	Permutation test	Identified *TYRP1* gene	[30]
28	Racing distance	50K	118 elite Thoroughbred racehorses divergent for race distance aptitude	Chi-square test	Bonferroni correction P_unadj_. = 1.61e^-9^; P_Bonf._ = 6.58e^-5^	Identified a significant 690 kb region on ECA18 containing *MSTN* gene	[31]
29	Dwarfism	50K	Ten Friesian dwarf horses vs ten controls	Chi-square test	Bonferroni correction *P <* 1.72e^-6^	Identified a significant region on ECA14: 3.8-5.4 Mb containing *PROP1* gene	[33]
30	Lavender Foal Syndrome (LFS)	50K	Egyptian Arabian including 7 affected foals, their 31 relatives, as well as 114 controls	Fisher’s exact test	*P* < 0.05	Identified a significant region containing *RAB27A* and *MYO5A* genes	[34]
31	Recurrent laryngeal neuropathy (RLN)	50K	234 cases (196 Warmbloods, 20 Trotters, 14 Thoroughbreds, and 4 Draft horses), 228 breed-matched controls	Chi-square test	Bonferroni correction *P <* 1.09e^-6^ (significant); *P <* 2.11e^-5^ (suggestive)	Identified two significant SNPs on ECA21 and ECA31	[35]
32	Horn morphology	50K	107 Soay sheep from the neighbouring island of Soay	Chi-square test	K_eff_ correction of *P <* 1.859e^-6^	Identified a significant region on Chr10 including *RXFP2* gene	[36]
33	Inherited Rickets	50K	Corriedale sheep including 17 affected and 3 carriers	IBD analysis	*P* < 0.05	Identified a 6Mb region on Chr6 including *DMP1* gene	[40]
34	Degenerative myelopathy (DM)	50K	Pembroke Welsh corgi including 38 DM-affected cases and 17 controls	Chi-square test	*P* < 0.01	Identified a region of 28.91-29.67 Mb on CFA31 including SOD1 gene	[43]
35	Canine atopic dermatitis (cAD)	20K	48 Golden Retrievers including 25 with atopic dermatitis and 23 healthy controls	Chi-square test	*P* < 0.001	Identified 35 significant SNPs	[46]
36	Arrhythmogenic right ventricular cardiomyopathy (ARVC)	50K	65 ARVC-affected boxer dogs vs 100 controls	Chi-square test	*P* < 0.05	Identified a region of CFA17: 32,256,760-32, 388,077bp containing *STRN* gene	[47]
37	Intervertebral Disc Calcification	20K	Dachshund dogs including 48 cases and 46 controls	Chi-square test	Permutation test using 100,000 permutations	Identified a region of CFA12: 36.8-38.6Mb with 36 significant SNPs	[48]
38	Fatness	3K	720 birds from two populations including F_2_: Broiler × Fayoumi and F_2_: Broiler × Leghorn	One-way ANOVA test	*P* < 0.01	Identified 39 significant SNPs mainly on GGA1, 2, 3, 4, 7, 8, 10, 12, 15 and 27	[49]
39	Body weight	60K	278 individuals from F_2_ population crossed by Silky Fowl × White Plymouth Rock	Linear regression analyses	Bonferroni correction *P <* 1.92e^-6^ (significant); *P <* 3.85e^-5^ (suggestive)	Identified 9 significant SNPs on GGA4: 71.6-80.2 Mb including *LDB2* gene	[50]
40	Growth traits	60K	489 birds from F_2_ population crossed by WRR × XH	Generalized least square analysis	Bonferroni correction *P <* 4.08e^-8^ (highly significant); *P <* 2.04e^-6^ (significant); *P <* 4.08e^-5^ (suggestive)	Identified 68 significant SNPs and 23 genes for 18 growth traits	[51]
41	Egg production and quality	60K	385 White leghorn and 361 brown-egg dwarf layers	Fisher’s combined probability method	Bonferroni correction *P <* 1.5 e^-6^,	Identified 8 significant SNPs and two genes including *GRB14* and *GALNT1*	[52]

### Cattles

More than ten papers described the use of GWAS for several economically important traits in cattle, including milk yield, milk quality, fertility, growth, meat quality and carcass traits, were reported. For milk yield in dairy cattle, there were four GWAS reports, and a total of 734 SNPs with significant effects on milk yield were detected [4-7]. These SNPs were mainly on chromosomes 8, 9, 10, 11, 13, 25 and 29 and a significant SNP was located close to the *DGAT1* gene (160bp apart). For the milk quality trait (eg. fatty acid composition, protein percentage, fat percentage), there were also four GWAS reports, and 547 SNPs on chromosomes 5, 6, 11, 14, 19 and 26 were significantly associated with milk quality [8-11]. The genes, identified from the GWAS results, that might be important for milk quality traits included *ABCG2PPARGC1AACSS2DGAT1ACLYSREBF1STAT5AGHFASNSCD1* and *AGPAT6*. Another four GWAS reported 198 significant SNPs related to the fertility trait such as fertilization rate, clastocyst rate and calving [12-15]. These SNPs were mainly on chromosomes 3, 4, 5, 6, 10, 12, 13, 18, 19, 20, 24 and 25, and the important genes detected from the GWAS results were collagen type I alpha 2 and integrin beta 5. The results indicated that the incubation of bull spermatozoa with antibodies against integrin beta 5 significantly decreased their ability to fertilize oocytes suggesting that the bovine sperm integrin beta 5 protein play an important role during fertilization and could serve as a positional or functional marker of fertility in the bull. Snelling et al. [16] and Bolormaa et al. [17], respectively, reported GWAS on the cattle growth trait (eg. body weight and height), and a total of 306 significant SNPs were detected. These significant SNPs were mainly on chromosomes 3, 5, 7 and 8. There has been only one GWAS study on cattle meat quality, reported by Bolormaa et al. [18]. In total, 940 beef cattle were used in this study and 87 SNPs with significant effects on meat quality (intramuscular fat percentage) were detected. This GWAS also detected 127 SNPs with significant effects on carcass traits (longissimus muscle and rump fat). Classical bovine spongiform encephalopathy (BSE) was a disease that invariably cause fatal in cattle and has been implicated as a significant human health risk. A GWAS on BSE was carried out using the SNP50 beadchip in Holstein cows [19]. The results of this study revealed that the a SNP on chromosome 1 at 29.15 Mb was associated with BSE disease and another locus on chromosome 14, within a cluster of SNPs showed a trend toward significance. The genes within these regions might be important for BSE and need to be further investigated. Bovine tuberculosis (TB) was a significant veterinary and financial problem in many parts of the world. Finlay et al. carried out a GWAS on bovine tuberculosis using Irish dairy herd and the results indicated that 3 SNPs in a 65kb genomic region on BTA 22 were significantly associated with tuberculosis susceptibility [20]. The *SLC6A6* gene within this region might be important for tuberculosis. Another GWAS report was also focused on tuberculosis using two populations of Holstein cows and 6 SNPs on chromosomes 1, 12 and 15 in one population and several SNPs on chromosomes 1, 6, 7, 13, 16, 21, 23 and 25 in another population were detected for their significant association with Paratuberculosis [21]. The genes related to these significant SNPs might be important for Paratuberculosis in cattle. The 770K SNP chip for Bovine was a high density (HD) bead array from Illumina, containing 777,000 SNP markers. This high density SNP chip allows a variety of applications including genome wide selection and identification of quantitative trait loci. Philipp et al. carried out a GWAS using this HD bead array in German Fleckvieh Cattle to detect the mutations associated with Dominant White Phenotype and Bilateral Deafness [22]. The results of this study revealed a most significantly associated region on bovine chromosome (BTA) 22. There were 13 genes in this significant region, including *MITF*, which was essential for the development and post-natal survival of melanocytes. The further sequence analysis of this gene revealed that there was a missense mutation in exon 7 that was associated with Dominant White Phenotype and Bilateral Deafness.

### Pigs

An example of a GWAS on androstenone levels in male pigs was reported by Duijvesteijn et al. [23]. They used the Illumina Porcine 60K SNP Beadchip and genotyped 987 pigs divergent for androstenone concentration from a commercial Duroc-based sire line. The association analysis, which involved 47,897 SNPs, revealed that androstenone levels in fat tissue were significantly affected by 37 SNPs mainly on porcine chromosomes 1 and 6. On chromosome 6, a large region of 10 Mb was shown to be associated with androstenone, and this region covered several candidate genes that are potentially involved in the synthesis and metabolism of androgens. The chromosome 6 might be an important chromosome in the determination of androstenone levels. Skatole is another component of boar taint, in addition to androstenone. Ramos et al. [24] carried out a GWAS for skatole using the same animals as Duijvesteijn et al. [23]. The results indicated that 16 SNPs located on the proximal region of chromosome 6 were significantly associated with skatole levels but no obvious candidate genes could be pinpointed in the region. Using GWAS and LDLA (linkage disequilibrium and linkage analysis) analysis, Grindflek et al. found 28 chromosome regions related to boar taint in commercial Landrace and Duroc breeds [25]. These chromosome regions were mainly on chromosomes 1, 2, 3, 5, 6, 7, 10, 11, 13, 14 and 15. Further study was carried out using 1,533 purebred Landrace and 1,027 purebred Duroc and a total of 34 regions were found significantly associated with boar taint and fertility traits. These 34 regions were mainly on chromosomes 1, 2, 3, 4, 7, 13, 14 and 15 [26].

Sironen et al. reported a GWAS on infertility (knobbed acrosome defect, KAD) trait in the Finnish Yorkshire pig population using the PorcineSNP60 Genotyping BeadChip, and the KAD-associated region was identified within 0.7 Mbp on porcine chromosome 15 [27]. There were two genes, *STK17b* and *HECW2*, located within this region. The sequencing in the protein coding region of these two genes revealed two SNPs within *HECW2* gene, but no polymorphisms were detected within *STK17b* gene. One nonsynonymous SNP identified within the *HECW2* gene was further genotyped for all 14 KAD-affected and 10 control boars. All KAD-affected boars were homozygous for this SNP, but also four control boars had the same homozygous allele, indicating that this SNP was unlikely to be the causal mutation.

Fan et al. used Illumina’s PorcineSNP60 BeadChip to perform a GWAS on 820 commercial female pigs that were phenotyped for backfat, loin muscle area and body conformation in addition to traits of foot and leg (FL) structural soundness [28]. A total of 51,385 SNPs were used in the GWAS and a number of candidate chromosomal regions were discovered; some of them corresponded to QTL regions reported previously. In these regions, some well-known candidate genes for the traits of interest were identified, such as *MC4R* (for backfat) and *IGF2* (for loin muscle area), and a number of novel promising genes were reported, including *CHCHD3* (for backfat), *BMP2* (for loin muscle area, body size and several FL structure traits), and some *HOXA* family genes (for overall leg action). Functional clustering analyses classified the genes into categories related to bone and cartilage development, muscle growth and development or the insulin pathway, which suggested that the traits were regulated by common pathways or gene networks that exert roles at different spatial and temporal stages.

Fatness is one of the important economic factors in pork production, and also associated with serious diseases in humans. Ponsuksili et al. applied a GWAS to traits of hepatic gene expression, focusing on transcripts with expression levels that correlated with fatness traits in a porcine model [29]. A total of 150 pigs were studied for transcript levels in the liver. The 24K Affymetrix expression microarrays and 60K Illumina single nucleotide polymorphism (SNP) chips were used in the study. A total of 663 genes, whose expression levels being significantly correlated with the trait “fat area”, were detected. The association between the genome-wide SNPs and expression of these 663 genes was analyzed and the result revealed 4,727 expression quantitative trait loci (eQTL).

Brown coat color is another important economic trait in pigs, and a GWAS was performed by Ren et al. using the Illumina PorcineSNP60 BeadChips on Tibetan and Kele pigs [30]. By means of a haplotype-sharing analysis, the critical region was refined to a 1.5-Mb interval on chromosome 1 that encompasses only one pigmentation gene: tyrosinase-related protein 1 (*TYRP1*). Mutation screens of sequence variants in the coding region of *TYRP1* revealed a strong candidate causative mutation (c.1484_1489del). The protein-altering deletion showed complete association with the brown coloration across Chinese-Tibetan, Kele, and Dahe breeds. It occurred exclusively in brown pigs and was absent from all non-brown-coated pigs from 27 different breeds. The findings provide compelling evidence that brown coloration in the three Chinese indigenous pig breeds is caused by the same ancestral mutation in *TYRP1*.

### Horses

It is widely recognized that inherited variation in physical and physiological characteristics of the horse is responsible for the variation in individual aptitude for racing distance, and that muscle phenotypes in particular are important. A genome-wide SNP-association study for optimum racing distance was performed using the EquineSNP50 Bead Chip genotyping array in a cohort of 118 elite Thoroughbred racehorses divergent for race distance aptitude [31]. The GWAS result indicated that the most significant SNP was located on chromosome 18 about 690 kb from the gene encoding myostatin (*MSTN*). Together with previous results [32], this indicated that the *MSTN* gene may be a major factor affecting racing distance in horses.

Dwarfism is also an important trait in horses. Orr et al. performed a GWAS on dwarfism in Friesian horses using 34,429 SNPs, and the most significant SNP was located close to a gene implicated in human dwarfism [33]. Lavender foal syndrome (LFS) is a lethal inherited disease of horses that has a suspected autosomal recessive mode of inheritance. Brooks et al. reported a GWAS for LFS using a small sample of 36 horses segregating for LFS [34]. These horses were genotyped using a newly available SNP chip containing 56,402 SNPs. The GWAS results indicated that the region containing two functional candidate genes encoding ras-associated protein RAB27a (*RAB27A*) and myosin Va (*MYO5A*) was significantly associated with LFS. Exon sequencing of the *MYO5A* gene from an affected foal revealed a single base deletion in exon 30. A PCR–RFLP result indicated that all affected horses were homozygous for this mutation. This locus might be the causal mutation for LFS in horses.

Another disease known as recurrent laryngeal neuropathy (RLN), is also important in horses. It causes abnormal respiratory noise during exercise and can impair performance. Dupuis et al. carried out a GWAS using the Illumina Equine SNP50 BeadChip in 234 cases (196 Warmbloods, 20 Trotters, 14 Thoroughbreds, and 4 Draft horses), 228 breed-matched controls, and 69 parents [35]. The result indicated that two loci reached suggestively significant level in Warmbloods, respectively on chromosomes 21 and 31. The two signals were driven by the enrichment of a “protective” haplotype in controls compared with cases. This result indicated that these two signals are important for RLN in horses.

### Sheep

The first report of the use of GWAS in sheep was made on horn types by Johnston et al. [36]. A genome-wide association study was conducted using 36,000 SNPs and determined the main genetic candidate for horns to be *RXFP2*, an autosomal gene with known involvement in determining primary sexual characteristics in humans and mice [37-39]. Evidence from additional SNPs in and around *RXFP2* supports a new model of horn-type inheritance in Soay sheep, and for the first time sheep with the same horn phenotype but different underlying genotypes can be identified. In addition, *RXFP2* was shown to be an additive quantitative trait locus (QTL) for horn size in normal-horned males, accounting for up to 76% of the additive genetic variation in this trait. This finding contrasts markedly with GWAS of quantitative traits in humans and some model species, where it is often observed that mapped loci only explain a modest proportion of the overall genetic variation.

The other study of GWAS in sheep was reported by Zhao et al. [40], who in the same year used the same Illumina OvineSNP50 BeadChip as Johnston et al. [36]. This study was focused on the inheritance of rickets in Corriedale sheep. A GWAS was carried out on 20 related sheep, comprising 17 affected individuals and 3 carriers. A homozygous region that included 125 consecutive SNP loci was identified in all 17 affected sheep, covering a region of 6 Mb on ovine chromosome 6. There were 35 genes in this region; the gene for dentin matrix protein 1 (*DMP1*) was sequenced and a nonsense mutation, 250C/T, was identified on exon 6. This mutation introduced a stop codon (R145X) and could truncate C-terminal amino acids. Genotyping by PCR–RFLP for this mutation showed that all 17 affected sheep had the “T T” genotype; the 3 carriers were “C T”; 24 phenotypically normal related sheep were either “C T” or “C C”; 46 unrelated normal control sheep from other breeds were all “C C”. The other SNPs in *DMP1* were not concordant with inherited rickets and can all be ruled out as candidates. Previous research has shown that mutations in the *DMP1* gene are responsible for autosomal recessive hypophosphatemic rickets in humans [41]. *Dmp1* knockout mice exhibit rickets phenotypes [42]. Therefore the R145X mutation in *DMP1* is thought to be responsible for inherited rickets in Corriedale sheep.

### Dogs

Degenerative myelopathy (DM) is a fatal neurodegenerative disease prevalent in several dog breeds. Awano et al. carried out a GWAS using 38 DM-affected Pembroke Welsh corgi cases and 17 related clinically normal controls [43]. This produced the strongest associations with markers on chromosome 31 in a region containing the canine *SOD1* gene. *SOD1* was considered to be a regional candidate gene from the results of previous studies in human and mice [44,45]. Re-sequencing of *SOD1* in normal and affected dogs revealed a G to A transition and homozygosity for the A allele was associated with DM in five dog breeds. The result indicated that the *SOD1* gene is important for DM in dogs.

Canine atopic dermatitis (cAD) is a common disease in dogs, and the first GWAS was reported by Wood et al. using the Illumina Canine SNP20 array [46]. The study used affected and unaffected Golden Retrievers to carry out the GWAS, and one SNP was over the log5 threshold and 35 SNPs were over the log3 threshold. Further validation studies of the top 40 SNPs from the GWAS results were performed using Sequenom genotyping of larger numbers of cases and controls across eight breeds. Two SNPs were associated with cAD in all breeds tested, and these two SNPs were located in intergenic regions. The effects of these two SNPs were independent of each other, indicating that further fine mapping and re-sequencing was required for these areas. Another 12 SNPs were shown by Sequenom genotyping to be associated with cAD, but these were not important in all breeds. The results of this study suggested that GWAS would be a useful approach to identify genetic risk factors for cAD.

Arrhythmogenic right ventricular cardiomyopathy (ARVC) is inherited most frequently as an autosomal dominant trait with incomplete age-related penetrance and variable clinical expression. A GWAS for ARVC was carried out by Meurs et al. using the canine 50k SNP array in adult Boxer dogs, which identified several regions significantly associated with ARVC, of which the strongest SNP resided on chromosome 17 [47]. Fine-mapping and direct DNA sequencing identified an eight base pair deletion in the 3' untranslated region (UTR) of the striatin (*STRN*) gene on chromosome 17 that was associated with ARVC in the Boxer dog. Further analysis indicated that the deletion affected a stem loop structure of the mRNA. Dogs that were homozygous for the deletion had a more severe form of disease, on the basis of a significantly higher number of ventricular premature complexes. The results of this study suggested that *STRN* may serve as a novel candidate gene for ARVC.

Intervertebral disc calcification and herniation commonly affect Dachshunds. The number of calcified discs at 2 years of age, determined by radiographic evaluation, is a good indicator of the severity of disc degeneration and thus serves as a measure of the risk of developing intervertebral disc herniation. A GWAS analysis was carried out to identify genetic variants associated with intervertebral disc calcification in Dachshunds [48]. In total, 48 cases with > =6 disc calcifications or that had been treated surgically for disc herniation and 46 controls with 0–1 disc calcifications were genotyped using the Illumina CanineHD BeadChip. A region on chromosome 12 from 36.8 to 38.6 Mb containing 36 significant SNPs was identified in the GWAS analysis. The results of this study suggested that the genetic variations in the region on chromosome 12 may be important for the development of intervertebral disc calcification in Dachshunds.

### Chickens

The first GWAS in chickens was reported by Abasht and Lamont using 3,000 SNPs on the whole genome in two F_2_ populations; the results indicated that there were 15 and 24 markers significantly associated (*P* < 0.01) with abdominal fatness (AF) in the two F_2_ populations, respectively [49]. These SNPs were on 10 chromosomes (1, 2, 3, 4, 7, 8, 10, 12, 15 and 27). Further analysis revealed that these SNPs were considered to be associated with QTL with cryptic alleles. This study revealed cryptic alleles to be an important factor in heterosis for fatness observed in two F_2_ populations of chickens, and suggested that epistasis was the common underlying mechanism for heterosis and cryptic allele expression.

There was a GWAS about chicken body weight [50]. A total of 26 SNP effects related to 9 different SNPs were significantly associated with body weight at 7–12 weeks of age. These significant SNPs were mainly in a region of the chicken chromosome 4 approximately 8.6 Mb in length (71.6–80.2 Mb). The LIM domain-binding factor 2 (*LDB2*) gene in this region had the strongest association with body weight for weeks 7–12, and with average daily gain for weeks 6–12. This gene may be important in the regulation of body weight in the chicken. Another GWAS about chicken growth was reported by Xie et al [51]. A total of 257 SNP effects involving 68 SNPs and 23 genes were detected for 18 traits with genome-wide significance [51]. Among these identified SNPs or regions, the 1.5 Mb region (173.5–175 Mb) of chicken chromosome (GGA) 1 was the most important for chicken growth traits and genes in this region may be important for chicken growth.

The egg production and quality traits were important in layer chickens. Liu et al. carried out a GWAS on chicken egg production and quality traits using two populations including White Leghorn and Brown-Egg Dwarf Layers. The result indicated that there were 8 SNPs significantly associated with egg production and quality traits [52]. Among these significant SNPs, several were located in known genes including *GRB14* and *GALNT1* that can impact the development and function of ovary.

## Conclusions

In summary, there was a great progress of GWAS in domestic animals and some genes for economically important traits have been identified. However, the main problem lies in the inconsistencies among the results of these GWAS reports for the same trait, which may be mainly attributed to many aspects such as population size, density of the markers (SNPs), population genetic structure, choice of statistical models, as well as type I and II errors. To achieve the accurate estimation of SNP effects on traits of interest in a GWAS, larger population size and higher density of the markers (SNPs) were required. Currently, SNP chips were widely applied in GWAS and enhanced the identification of QTL for traits of interest in domestic animals. Compared with SNP chips, sequencing could provide nearly all information about the variations, including SNP, copy number variation (CNV) and the deletion/insertion, et al., on the whole genome in detected population. Along with the reduction in sequencing cost, it is possible that all individuals in the tested populations might be sequenced and genotyped and GWAS might be carried out in this platform then. In the future, GWAS in domestic animals will focus on the identification of causative mutations for economically important traits. The findings will inevitably facilitate the understanding of the genetic architecture of complex traits in domestic animals and practical improving the breeding programmes.

## Abbreviations

QTL, Quantitative trait loci; GWAS, Genome wide association study; SNP, Single-nucleotide polymorphism; CI, Confidence interval; LD, Linkage disequilibrium; LDLA, Linkage disequilibrium and linkage analysis; KAD, Knobbed acrosome defect; FL, Foot and leg; eQTL, Expression quantitative trait loci; LFS, Lavender foal syndrome; RLN, Recurrent laryngeal neuropathy; DM, Degenerative myelopathy; cAD, Canine atopic dermatitis; ARVC, Arrhythmogenic right ventricular cardiomyopathy; AF, Abdominal fatness; CNV, Copy number variation.

## Competing interests

The authors declare that they have no competing interests

## Authors’ contributions

HZ collected the information used in the manuscript and drafted the manuscript. ZW collected the information and helped to draft the manuscript. SW collected the information and helped to draft the manuscript. HL co-led the conception and design of the study, participated in the collection of the information and contributed to writing the manuscript. All authors read and approved the final manuscript.
